# Characteristics of hydraulic fracture surface based on 3D scanning technology

**DOI:** 10.1098/rsos.171845

**Published:** 2018-06-20

**Authors:** Fan Zhang, Geng Ma, Yunqi Tao, Xiao Liu, Yixin Liu, Rui Li

**Affiliations:** 1 School of Energy Science and Engineering, Henan Polytechnic University, Jiaozuo, Henan 454003, People's Republic of China; 2 State Key Laboratory for Coal Mine Disaster Dynamics and Control, Chongqing University, Chongqing 400044, People's Republic of China; 3 Applied Technical College, China University of Mining and Technology, Xuzhou, Jiangsu 221008, People's Republic of China

**Keywords:** surface characteristic, hydraulic fracturing, 3D scanning, 3D coordinates, superficial area

## Abstract

The surface characteristics of fractured specimens are important in hydraulic fracturing laboratory experiments. In this paper, we present a three-dimensional (3D) scanning device assembled to study these surface characteristics. Cube-shaped rock specimens were produced in the laboratory and subjected to triaxial loading until the specimen split in two in a hydraulic fracturing experiment. Each fractured specimen was placed on a rotating platform and scanned to produce 3D superficial coordinates of the surface of the fractured specimen. The scanned data were processed to produce high-precision digital images of the fractured model, a surface contour map and accurate values of the superficial area and specimen volume. The images produced by processing the 3D scanner data provided detailed information on the morphology of the fractured surface and mechanism of fracture propagation. High-precision 3D mapping of the fractured surfaces is essential for quantitative analysis of fractured specimens. The 3D scanning technology presented here is an important tool for the study of fracture characteristics in hydraulic fracturing experiments.

## 1. Introduction

Hydraulic fracturing is an effective method for coalbed methane (CBM) drainage that is widely used in coal mines globally [1]. Hydraulic fracturing is influenced by multiple factors, including *in situ* stress in a coal seam, natural fractures, mechanical parameters of coal rock and flow rate [2–5]. The main fracture propagates parallel to the direction of maximum horizontal stress. There are different types of natural fractures in coal seams, these cause anisotropy and discontinuity in the coal rock and greatly affect the deformation and mechanical strength of coal rock, permeability of CBM reservoirs and fracture network [6]. The mechanical parameters of coal rock are the basis for studying the mechanism of hydraulic fracturing in CBM reservoirs.

A hydraulic fracturing experiment is an effective method to study the efficiency and mechanism of hydraulic fracturing [7]. Such experiments can monitor hydraulic fracturing visually and over time. Many studies have focused on fracture morphology and mechanism of propagation [8]. Experimental devices for monitoring hydraulic fracturing include computed tomography (CT) scanning, tracer agents, digital photography, acoustic emission and microscopic observation [9–12]. Zou *et al.* [9] found that CT scanning was an effective method for revealing fracture geometry in natural bedding developed shale; CT scan images could display directly the fracture network in fractured shale. Ishida [10] conducted hydraulic fracturing experiments by granitic rock specimens with different grain sizes and found that shear fracturing or tensile fracturing played different roles in fracture propagation processes through acoustic emission. Moreover, acoustic emission was monitored by a borehole sonde in field fracturing to measure rock stress. Stanchits *et al.* [11] carried out hydraulic fracturing experiments by means of sandstone under conditions of different injection rates and fluid viscosity; monitoring of acoustic emission could indicate the development of fractures. Chen *et al.* [12] conducted hydraulic fracturing experiments to study the effect of fluid viscosity on fracture propagation and fractures were microscopically observed via a fluorescent method.

Besides, when fracturing fluid is flowing in a specimen, the structure and roughness of the fractured specimen directly affect the fracture morphology and propagation [13,14]. However, the processes related to fracture morphology and mechanism of fracture propagation are not well understood, and relevant research on the roughness and structure of fractured specimens is scarce. There are difficulties in accurately monitoring the superficial structure and roughness of fractured specimens using existing monitoring equipment. Moreover, studies on the characteristics of fractured specimens lack qualitative descriptions and are short of quantitative analysis. Therefore, it is important to develop an effective device that can extract the characteristics of fractured rock specimens. In this article, a three-dimensional (3D) scanning device is used to scan a fractured rock specimen, based on the scanned data the following characteristics of the fractured specimen are extracted: 3D coordinates, superficial area, volume, shaded relief image, 3D scanned image and contour map. Compared with digital photos, the characteristics extracted from the fractured specimen using the 3D scanner provide clearer and more detailed observations of the structure, roughness and variations of the fractured surface. The technique presented in this paper can be used to obtain quantitative information of specimens in hydraulic fracturing experiments.

## 2. Description of hydraulic fracturing experimental device

### 2.1. Device for three-dimensional scanning of coal rock specimens

The main components of the 3D scanning device are two OKIO-B non-contact 3D scanners, a rotating platform (figure 1) and 3D scanning software. The device performs fast non-contact scanning and provides 3D coordinates of the scanned object. A 3D model of the surface of the fractured specimen is produced and displayed automatically based on the high-precision extracted 3D coordinates.

**Figure 1.** 3D scanning device for coal rock specimen.

Compared with CT scanning, the device has the advantages of low cost and short experiment time. The 3D scanning image of the target can be observed in real time during the scanning process. The OKIO-B non-contact 3D scanner is easy to operate and has a high-precision charge-coupled device sensor, which has been widely applied to industrial and geotechnical engineering. The 3D scanning precision ranges from 0.01 to 0.02 mm and the 3D scanning average distance ranges from 0.07 to 0.15 mm.

After hydraulic fracturing, the fractured specimen is placed on a rotating platform for non-contact 3D scanning to obtain the structure, roughness and other characteristics of the fractured specimen. As the specimen is made of cement, gypsum and pulverized coal, there will be black spots upon the surface of the fractured specimen. Black spots on the surface of the fractured specimen will result in blanks in the 3D model. Because the black spots cannot be scanned to form a 3D model, dye penetrant inspection materials are used on the specimen to fill these blanks.

### 2.2. Hydraulic fracturing experimental system

The hydraulic fracturing system is composed of a true triaxial hydraulic fracturing device, fracturing pump system, data collection system and other components, as shown in figure 2.

**Figure 2.** Hydraulic fracturing experimental system: (*a*) true triaxial hydraulic fracturing device, and (*b*) fracturing pump system.

The true triaxial hydraulic fracturing device (figure 2*a*) consists of a stiff frame, hydraulic jack, steel plate and steel tube. A cube specimen is placed on the stiff frame. Specific stresses are applied to the specimen by hydraulic jacks. The maximum loading range is 100 kN, the value of the applied stress is displayed on the metre installed on the hydraulic jack. The directions of maximum horizontal stress (*σ*_H_), minimum horizontal stress (*σ*_h_) and vertical stress (*σ*_v_) are shown in figure 2*a*. The specimen is held in the stiff frame by steel plates, the relevant stresses are applied gradually and uniformly according to the designed experiment programme. Steel tubes are installed between the steel plates and stiff frame to ensure the stability and balance of the cube specimen.

The fracturing pump system (figure 2*b*) consists of a servo supercharger, water tank and control valve, which are controlled by specific software. The fracturing fluid can be pumped at a rate of displacement or pressure, its maximum water pressure is 60 MPa. The water pressure and flow rate of fracturing fluid are digitally monitored and displayed on the computer screen. The data collection system is composed of a pressure sensor connected to the fracturing pump system controlled by the True Triaxial Testaid software. The data (injection time, water pressure and flow rate) can be saved in real time. Red fracturing fluid was used as a tracer agent to observe the fracture propagation pattern.

## 3. Example tests

### 3.1. Specimens

The identical cube specimens (figure 3) were of dimensions 200 × 200 × 200 mm and made of cement, gypsum and pulverized coal. The coal rock was collected from coal seam no. 4 of the Xintian Coal Mine in Guizhou province, China. Its uniaxial compressive strength is 8.53 MPa, tensile strength is 0.63 MPa, elastic modulus is 0.82 GPa, Poisson's ratio is 0.28 and firmness coefficient (Protodayakonov's coefficient) is 0.80. To make the mechanical parameters of coal rock close to those of similar materials an experimental programme is designed to study the mechanical parameters of similar materials. After a series of ratio tests, a ratio (the proportion of cement, gypsum, pulverized coal was 2 : 1 : 1) was chosen to form the cube specimens. The material was tested to obtain its mechanical parameters, which were close to those of coal rock. The test yielded a compressive strength of 5.38 MPa, tensile strength of 0.60 MPa, elastic modulus of 0.78 GPa, Poisson's ratio of 0.25 and firmness coefficient of 0.82.

**Figure 3.** Cube specimens made of similar materials.

### 3.2. Characteristics of the fractured surface

A cube specimen was placed under a horizontal stress difference of 1.50 MPa, the fracturing fluid rate is 3.2 ml s^−1^ and the characteristics of the fractured specimen were analysed by the 3D scanning device, as shown in figure 4.

**Figure 4.** Fractured specimen showing ‘red zone’ indicting fluid propagation path.

The flow path of fracturing fluid can be inferred from the red zone on the fractured specimen, as shown in figure 4. We can deduce the fracture morphology and propagation from the digital photo. The black spots on the fractured surface cannot be accurately scanned; therefore, they are filled with dye penetrant inspection material before scanning. To obtain a full set of 3D data points of the fractured surface, the specimen is placed under the OKIO-B non-contact high-precision 3D scanner on a continuously rotating platform. The scanned data are processed automatically to produce the 3D model.

Figure 4 shows that the fracture propagates perpendicular to the direction of minimum horizontal stress. The characteristics of the fractured surface, including the shaded relief model, 3D scanning image, contour map, superficial area, volume and 3D coordinates, can be derived by the 3D scanning device.

Compared with the digital photograph of the fractured specimen (figure 5*a*), the 3D shaded relief image (figure 5*b*) produced by the 3D scanner presents a much clearer view of the variation and roughness of fractured surface. The 3D coloured scanning image (figure 5*c*) illustrates the fine structural details of the fractured surface. The contour map of the fractured surface is shown in figure 5*d*, the areas where the contour lines are close together represent a more complex fracture pattern, where the dynamic effect of the fracturing fluid is stronger and the flow rate is higher. Based on the 3D coordinate dataset, the superficial area of fractured surface and volume of fractured specimen are 41820.67 mm^2^ and 3317200.78 mm^3^, respectively.

**Figure 5.** 3D imaging and map produced by the 3D scanner: (*a*) digital image of the fractured specimen; (*b*) shaded relief model of the fractured specimen; (*c*) 3D scanning image of the fractured specimen; and (*d*) contour map of the fractured specimen.

## 4. Conclusion

A 3D scanning device was used to scan the surface of fractured rock specimens and extract the surface characteristics. The specimens were fractured in a hydraulic fracturing experiment. The scanned data were processed to produce a shaded relief model of the fractured specimen, a 3D scanning image and a contour map of the fractured surface, generating a clear and detailed representation of the fracture morphology and propagation. A new method is proposed to quantitatively study hydraulic fracturing. Using the 3D coordinates extracted from the scanner, the superficial area of the fractured surface and volume of the fractured specimen can be derived for quantitative analysis. The 3D scanning device for coal rock specimens is an efficient diagnostic tool for hydraulic fracture experiments.

## Supplementary Material

Data for producing Figure 5c and d

## Supplementary Material

Data of superficial area and volume of fractured specimen

## Supplementary Material

Data for producing Figure 5b

## Data accessibility

The data can be accessed in the electronic supplementary material.
